The article "Application of Expert Adjustable Fuzzy Control Algorithm in Temperature Control System of Injection Machines" was retracted in 2023. Reasons: unreliable results or conclusions; concerns about the data; concerns about the results or conclusions; concerns about the peer review.

# Application of Expert Adjustable Fuzzy Control Algorithm in Temperature Control System of Injection Machines

**DOI:** 10.1155/2022/3616814

**Published:** 2022-06-27

**Authors:** Yanan Hu, Kun Wu

**Affiliations:** Xijing University, Xi'an 710000, China

## Abstract

The stability and accuracy of temperature control of the injection molding machine is one of the keys to determine the quality and appearance of plastic parts. Due to the temperature control system of water-cooled injection molding machine has the characteristics of coupling, nonlinearity, and hysteresis, the traditional proportion-integral-derivative (PID) method to control the barrel temperature of injection molding machine will yield temperature overshoot and oscillation, affecting the product and appearance quality. In order to improve the effect of barrel temperature control, in this paper, an expert adjustable fuzzy control strategy (EAFCA) is designed to optimize the barrel temperature control system through the combination of expert control, fuzzy control, and PID control. The expert control rules are designed according to the barrel temperature deviation *e* and its change rate ec. The expert rules are used to adjust the mapping range of the fuzzy universe in real time for the input and output variables of the fuzzy controller and finally to realize the accurate adjustment of the PID controller parameters. In terms of control systems, the distributed control system (DCS) monitoring system of injection molding machine is designed with Siemens CPU315-2PN/DP and industrial computer as the hardware core and Step7 and windows control center (WinCC) as the software platform to complete the tool plastic production monitoring system. The DCS improves the operability, data management convenience, and plastic production efficiency of the injection molding machine monitoring system. The Simulink simulation and field test show that the EAFCA method can increase the adjustment speed by approximately 34 s and reduce the overshoot by nearly 3.1%, which significantly improves the stability and accuracy of the barrel temperature and improves the quality of plastic parts.

## 1. Introduction

With the development of science and the reduction of plastic production costs, engineering plastics are widely used in electronics, aerospace, medical and health, automobile manufacturing, and other industries, and the demand is steadily rising [1–3]. Water-cooled injection machines perform well in cooling speed, production efficiency, and qualities of plastic parts and are widely used in the manufacturing of plastic parts. The effect of temperature control of injection machines is a key link in production quality and appearance [4–6]. Compared to traditional injection machines, water-cooled injection machines have more complex control systems. The barrel temperature is not only affected by the friction between plastics, the coupling between neighborhood temperature fields, and voltage fluctuation [7] but also influenced by the temperature and flow rate of cold circulating water, which may result in temperature oscillation and poor stability of barrel and further reduce the quality of plastic products and the service life of the equipment [8].

The article "Application of Expert Adjustable Fuzzy Control Algorithm in Temperature Control System of Injection Machines" was retracted in 2023. Reasons: unreliable results or conclusions; concerns about the data; concerns about the results or conclusions; concerns about the peer review.

At present, the single interval proportion-integral-derivative (PID) controller is usually used to control the barrel temperature of injection machines, which ignores the needs of barrel temperature control with coupling, nonlinearity, and complexity [9, 10]. To address these problems, some scholars have proposed to use Smith predictor to improve the hysteretic system in related fields but not considered the nonlinear and coupling [11–13]. Furthermore, a genetic-simulated annealing algorithm (GSAA) was proposed to optimize the barrel temperature control system [14]. GSAA integrated the local optimization ability of the simulated annealing algorithm and the global search ability of the genetic algorithm to reduce the overshoot and the adjustment time of barrel temperature. However, GSAA is too complex to implement, and it requires high-grade hardware configuration of the computer system [15–17]. Other scholars adopted fuzzy control to adjust the parameters of PID controllers but ignored the limitation of the fixed domain of fuzzy control rules [18–20].

The fuzzy PID controller is widely applied to the process control system with complex working conditions, the controlled object model which is hard to solve and high control precision, because it is advanced, simple, and easy to implement. Based on the fuzzy control rule library and fuzzy inference machines, the parameters of the PID controller can be set online in real time and the PID controller becomes dynamic, flexible, and intelligent, which is superior to the phenomenon that traditional PID controller cannot adapt to the time-varying environment with much interference. Expert control can adjust the range of variable universe of fuzzy control rules according to the expert control rules in the knowledge base. The mapping range of fuzzy universe is adjusted, without increasing the number of fuzzy control rules. EAFCA is designed to improve the control accuracy of the system by adjusting the variable domain of fuzzy PID through expert control, which can break through the contradiction between accuracy of the traditional fuzzy PID control and the complexity of the controller and the fine of fuzzy rules.

The article "Application of Expert Adjustable Fuzzy Control Algorithm in Temperature Control System of Injection Machines" was retracted in 2023. Reasons: unreliable results or conclusions; concerns about the data; concerns about the results or conclusions; concerns about the peer review.

In this paper, a temperature control scheme of injection molding machine, namely, the EAFCA is proposed. In the aspect of control algorithm, according to the expert knowledge and field control requirements, the expert knowledge base for adjusting the domain of fuzzy variables and the fuzzy PID control rules for temperature regulation are designed and then EAFCA is constructed to solve the problem of low short-time control accuracy caused by the fixed domain of fuzzy variables. The algorithm makes use of the advantage of fuzzy PID in nonlinear and time-varying control systems. Simulink software simulation: EAFCA improves the accuracy of the barrel temperature control system. The control system is designed based on CPU315-2PN/DP controller and industrial computer as hardware, Siemens Step7 and Windows Control Center (WinCC) as the software development platform, and Profinet as the communication protocol. This paper completes the hardware selection, program design, and human machine interface (HMI) development and realizes the distributed control system (DCS) of injection molding machine to improve the equipment production efficiency, plastic product quality, and workshop automation level.

## 2. The Principle of Barrel Temperature Control

The barrel temperature control system of water-cooled injection machines mainly includes CPU315-2PN/DP controller, SM331 analog input module, SM332 analog output module, and SM322 digital output module, temperature sensor, heating wire, electromagnetic control valve, solid state relay (SSR), touch screen, and industrial computer.

The temperature control principle of the barrel is shown in Figure 1. PT100 thermistor is selected as the temperature sensor of injection molding machine. Its model is SBWZ, the temperature range is 0∼300°C, and the output signal is 4∼20 mA. The three PT100 temperature sensors located on the outer wall of the barrel detect the real-time temperature and simultaneously convert the temperature signal into a standard current signal of 4 ∼ 20 mA, which is transmitted to SM331 module. SM331 performs A/D conversion, then converts the standard current signal to 0 ∼ 27648 digital signal, and sends it to CPU315-2PN/DP controller. CPU315-2PN/DP carries out logical operation and conditional operation according to the project functional program Step7 and transfers the operation results to the SM332 or SM322 output module in the form of instructions, so as to control the action of the heating wire or the electromagnetic regulating valve and realize the heating or cooling of the barrel. When the temperature process value (PV) is lower than the set point (SP), control program unit (CPU) outputs the ratio of turn-on and turn-off of SSR. SM322 adjusts the heating wire power to increase the temperature of barrel; when the PV value is higher than the SP value, the large thermal inertia of the injection machines in the heating process causes temperature overshoot. Then, the CPU outputs control quantity, the SM332 outputs a standard current of 4 ∼ 20 mA to adjust the valve opening of the solenoid valve for cooling circulating water, and the cooling water is introduced to cool the barrel temperature, so as to avoid the long adjustment time and slow speed of the temperature overshoot.

The article "Application of Expert Adjustable Fuzzy Control Algorithm in Temperature Control System of Injection Machines" was retracted in 2023. Reasons: unreliable results or conclusions; concerns about the data; concerns about the results or conclusions; concerns about the peer review.

## 3. The Design of EAFCA

### 3.1. Fuzzy PID Controller

In the fuzzy PID controller for barrel temperature of injection machines, the temperature deviation of barrel *e* and its change rate ec are taken as input variables; while the variation of the basic three parameters of PID controller are taken as output variables. It avoids short-term and large-scale fluctuations in the input signal caused by the distortion of the temperature control system, the fluctuation of the temperature detection signal, etc. It further avoids the shock of barrel temperature caused by instantaneous excessive adjustment of the output control quantity of the controller. Therefore, the real-time parameters P (proportion), I (integral), and *D* (differential) consist of two parts: fixed parameters and adjusting parameters.

(1) $$\begin{array}{c} \left\{\begin{array}{c} K_{P}=K_{P0}+\Delta K_{P}\\ K_{I}=K_{I0}+\Delta K_{I}.\\ K_{D}=K_{D0}+\Delta K_{D} \end{array}\right.. \end{array}$$

For formula (1), *K*_*P*_, *K*_*I*_, and *K*_*D*_ are real-time parameters; *K*_*P*0_, *K*_*I*0_, and *K*_*D*0_ are fixed parameters; and Δ*K*_*P*_, Δ*K*_*I*_, and Δ*K*_*D*_ are adjusting parameters.

Through summing up along with analysis, the adjustment experience of parameters in the barrel temperature control system and the expert knowledge in related control fields can be acquired. Then, scientific and reasonable fuzzy rules during PID parameters adjustment for barrel temperature control can be formulated in line with site requirements. Set the fuzzy subsets of input and output variables *e*, ec, Δ*K*_*P*_, Δ*K*_*I*_, and Δ*K*_*D*_ as NB (negative big), NM (negative medium), NS (negative small), Z (zero), PS (positive small), PM (positive middle), and PB (positive big). The parameters of the fuzzy PID controller are shown in Table 1. Since the temperature control of the barrel is accomplished by the cooperation of the heating device and the cold circulating water device, the switching threshold (*y*) is set to prevent frequent switching between the temperature control system devices to avoid the shock of the system. *w* is the parameter of the system regulation device. When *w* > 0, the cold circulating water device starts to rapidly cool down the barrel; while when *w* < 0, it will dissipate heat in a natural way. Therefore, two temperature adjustment devices should simultaneously be considered in the design of fuzzy control rules. The fuzzy input and output quantities are determined in the way of “IF *e* is…AND ec is…THEN … Δ*K*_*P*_ is… Δ*K*_*D*_ is… Δ*K*_*I*_ is … . After superposition and optimization of all the relationship rules, 49 fuzzy control rules are obtained to complete the formulation of fuzzy control rules, as shown in Table 2.

The article "Application of Expert Adjustable Fuzzy Control Algorithm in Temperature Control System of Injection Machines" was retracted in 2023. Reasons: unreliable results or conclusions; concerns about the data; concerns about the results or conclusions; concerns about the peer review.

The fuzzy PID adjustment rule of the barrel temperature is as follows: (1) When the positive direction of temperature *e* and ec is larger, larger Δ*K*_*P*_, smaller Δ*K*_*D*_, and smaller Δ*K*_*I*_ are selected to improve the response speed of cooling water valve for rapid cooling and prevent system differential and overshoot. (2) When the temperature *e* and ec are both positive and medium, appropriate Δ*K*_*P*_ and Δ*K*_*I*_ values are selected to ensure the proper response speed of the cooling system and prevent integral saturation. (3) When the temperature *e* is positive larger and ec is negative larger, appropriate Δ*K*_*D*_ and Δ*K*_*I*_ are selected to ensure appropriate response speed and prevent overshoot.(4) When the temperature *e* is positive larger and ec is negative smaller, the values of Δ*K*_*P*_ and Δ*K*_*D*_ should be appropriately reduced. (5) When the temperature *e* is positive smaller and ec is negative larger, reduce Δ*K*_*P*_ and increase Δ*K*_*D*_ to prevent system overshoot. (6) When the temperature *e* is positive smaller and ec is negative smaller, reduce Δ*K*_*P*_ and increase Δ*K*_*D*_ to prevent system overshoot. (7) When the temperature *e* and ec are both larger in the negative direction, select larger Δ*K*_*P*_, smaller Δ*K*_*D*_, and smaller Δ*K*_*I*_ to increase the SSR cut-off ratio for rapid heating. (8) When the temperature *e* and ec are both negative and medium, appropriate Δ*K*_*P*_ and Δ*K*_*I*_ values are selected to ensure the appropriate response speed of the heating system and prevent integral saturation. (10) When the temperature *e* is negative larger and ec is positive larger, properly reduce Δ*K*_*P*_ and increase Δ*K*_*D*_ to prevent system overshoot. (11) When the temperature *e* is negative smaller and ec is positive larger, it should decrease Δ*K*_*P*_ and increase Δ*K*_*D*_ and Δ*K*_*I*_. (12) When the temperature *e* is negative smaller and ec is positive smaller, reduce Δ*K*_*P*_ and increase Δ*K*_*D*_ and Δ*K*_*I*_ to prevent system overshoot. (13) In other cases, the values of Δ*K*_*P*_, Δ*K*_*D*_, and Δ*K*_*I*_ shall be adjusted appropriately according to the control requirements. The adjustment rules of PID fuzzy control parameters are shown in Table 2.

The article "Application of Expert Adjustable Fuzzy Control Algorithm in Temperature Control System of Injection Machines" was retracted in 2023. Reasons: unreliable results or conclusions; concerns about the data; concerns about the results or conclusions; concerns about the peer review.

### 3.2. Expert Adjustable Fuzzy Domain

Fuzzy PID controller can adjust the parameters online in real time, but the domain of variables is fixed in traditional fuzzy controller, which makes it difficult to respond the linguistic variable and fuzzy rules during the output of the optimal parameters. Expert control is a kind of intelligent control based on knowledge, and the control rules are not limited by control objects and criterion. The domain of fuzzy variables can be adjusted according to expert knowledge. Compared to the methods of function, neural network, and fuzzy control, the expert control algorithm has the advantages of simpler design, less difficulty in implementation, and convenient human-computer interaction. The barrel temperature control system adopting expert adjustable fuzzy-domain PID controller for injection machines is shown in Figure 2.

By Figure 2, the barrel temperature control system for injection machines adopts three-layer controller and dual-regulation device. The structure of three-layer controller is as follows: (1) The first layer is the expert adjustable fuzzy domain unit; the temperature sensors detect the real-time temperature of the barrel SP and send the converted signals of SP to CPU315–2PN/DP. Then, numerical and logical operations will be performed to acquire the values of *e* and ec which will be sent to the knowledge base and inference engine controlled by experts. The inference engine adopts forward reasoning method to discriminate each rule successively and get the optimal adjustment coefficient *a*(*e*), Ψ(ec), and *β*(pid) of fuzzy domain. The empirical rule set is a summary of control mode and control experience for the barrel temperature. Through the HMI interface, the control rules can be created, deleted, and modified to facilitate the update of the control rules and improve the flexibility of the combined application of expert knowledge. (2) The second layer is the fuzzy control unit. It takes the values of *e* and ec as the input variables and, at the same time, receives the optimal domain adjustment coefficient of fuzzy variables from the first layer. Then, the fuzzy inference will be performed according to the current domain scope to obtain the adjustment parameters Δ*K*_*P*_, Δ*K*_*I*_, and Δ*K*_*D*_, which can be added to the fixed parameters *K*_*P*0_, *K*_*I*0_, and *K*_*D*0_, respectively. The real-time parameters can be acquired. (3) The third layer is the temperature adjustment unit. The PID controller adjusts the output signals of the barrel temperature control system based on the real-time parameters. After calculating the value *e* and *y* to get the adjustment parameter *w*, Step7 starts to control the action of heating wire/cold circulating water, and then the barrel temperature will increase/decrease as the system needs. Barrel temperature is adjusted accurately and rapidly. The functions of the dual-regulation device are as follows: (i) The barrel heating device mainly consists of SSR, heating wire, SM322, etc. CPU outputs the turn-on and turn-off of the ratio of SSR. SM322 adjusts the heating wire power to increase the temperature of the barrel. (ii) The barrel cooling device mainly consists of electromagnetic valve, SM332, cold circulating water device, etc. The valve opening of solenoid valve is obtained by logic operation of CPU315–2PN/DP. After the D/A signal conversion, SM332 adjusts the valve position to change the flow of cold circulating water into the barrel. In this way, the barrel temperature will be reduced, and what must be noted here is to prevent overshoot.

The article "Application of Expert Adjustable Fuzzy Control Algorithm in Temperature Control System of Injection Machines" was retracted in 2023. Reasons: unreliable results or conclusions; concerns about the data; concerns about the results or conclusions; concerns about the peer review.

## 4. The Design of Control System for DCS

### 4.1. Hardware Selection

Generally, the traditional injection machines are controlled by the relay circuit, which causes low accuracy, high failure frequency, and low qualification rate. While DCS can realize distributed control, centralized operation, remote management, flexible configuration, and convenient configuration, CPU315-2PN/DP PLC integrates Profinet communication function. It can directly build a communication network with industrial computer and touch screen without adding a communication function module. It has the advantages of good economy, convenient operation, and easy maintenance. Siemens SM300 series modules have the characteristics of small size, fast speed, standardization, high reliability, convenient installation, and easy maintenance. KTP1000 has the advantages of convenient installation, flexible operation, friendly interface, and good compatibility, which is convenient for field personnel to control the equipment and modify parameters. Taking CPU315-2PN/DP PLC, touch screen, and industrial PC as the core of hardware, the SM module is integrated in the control system of DCS to achieve the close loop control on-site.

Through analyzing the needs of process, control, and maintenance for the control system of DCS, the hardware model can be selected. As shown in Figure 3, Siemens TIA selection tool can be used to simulate hardware installation and communication of the control cabinet to ensure the accuracy of module quantity, accessories, models, order number, and other information. It avoids the problems of the deviation of module number, model errors, communication failures, etc. The hardware selection of the control system of DCS is listed in Table 3.

The article "Application of Expert Adjustable Fuzzy Control Algorithm in Temperature Control System of Injection Machines" was retracted in 2023. Reasons: unreliable results or conclusions; concerns about the data; concerns about the results or conclusions; concerns about the peer review.

### 4.2. Program Design

The program of the control system for DCS is developed on the Step7 software platform. Based on the idea of modular programming, the main program calls each function program and interrupts the program to control the logic, sequence, and selection of injection machines. The temperature control of injection machines is divided into three sections, including solid conveying section, compression section, and metering section, and their control logic program is written in OB101, OB102, and OB103 tissue blocks, respectively. As shown in Figure 4, the control system begins to initialize after CPU315-2PN/DP PLC is powered on. Then, the initial parameters of PID, fuzzy control, and field control can be set. The temperature PV value is acquired through sampling and filtering program and is stored in DB200 data block. The comparison function program is called by CPU315–2PN/DP to compare DB200 and DB202 (SP value), and the results are stored in DB204 data block (*e* value). Then, we branch the program according to the value in DB204. When the value is not equal to 0, the ec value is calculated and stored in DB206. Expert control OB150 will receive the two data interfaces DB204 and DB206 and will obtain the optimal fuzzy domain coefficient using the reasoning function of the program and expert base. The above coefficient is stored in DB210∼DB218. Subsequently, the values in DB204, DB206, and DB210∼DB218 will be transmitted to the program of fuzzy control. By looking up the table of fuzzy control rule, the PID adjustment parameters Δ*K*_*P*_, Δ*K*_*I*_, and Δ*K*_*D*_ are obtained and then stored in DB210～DB218 data block. Sum of the PID fixed parameter values is stored in DB100∼DB104 and the PID adjustment parameter values are stored in DB300∼DB304, and the results are stored in DB450∼DB454 data blocks. According to the real-time data and the values of DB204 and DB206, the PID controller performs logic operations to get the control signals and stores it in DB208. If the value in DB204 is bigger than that in DB210 (threshold), the control signal will be converted to D/A by SM332, and the opening of solenoid valve is adjusted to cool the barrel; otherwise, the control signals adjust the turn-on and turn-off ratio of SSR by SM322 and change the heating wire power. Finally, the action of heating or natural cooling is carried out, and the accuracy control of the barrel temperature is achieved.

### 4.3. The Design of HMI Interface

HMI interface is a channel of human-machine interaction for centralized operation and remote management of the DCS. User login, fault alarm, production report, process flow, and other interfaces are designed based on WinCC platform. Advantages of DCS control system operability of injection molding machine are as follows: (1) Convenient operation process: it mainly monitors and controls the production process of the injection molding machine through the operator station, integrates the display function, process monitoring function, remote control function, and data storage and analysis function, and improves the convenience of operation and management security. (2) Easy software development: WinCC has built-in operation and management functions, which has the advantages of efficient configuration, simple integration and design, and flexible configuration and can develop the personalized operating system according to the control and operation requirements. (3) High operation efficiency: DCS can quickly complete data collection and centralized display, which can save data statistics time and reduce talent cost. As shown in Figure 5, the process flow interface of the injection molding machine DCS monitoring system can visually display the core parameters and process data of the injection molding process. Users can remotely view the temperature, value opening, heating state, motor state, and injection pressure of the on-site injection machines. The parameter setting interface can set and modify production parameters in a centralized and efficient manner. The historical curve interface can directly, quickly, and accurately query important parameters and monitored object data, which is conducive to alarm fault diagnosis and troubleshooting. The production report interface can record the generation time, quantity, model, and other information of plastic parts, which is convenient for production process management. To sum up, the injection molding machine DCS monitoring system realizes the centralized management, efficient operation, and integrated operation of the injection molding production process.

The article "Application of Expert Adjustable Fuzzy Control Algorithm in Temperature Control System of Injection Machines" was retracted in 2023. Reasons: unreliable results or conclusions; concerns about the data; concerns about the results or conclusions; concerns about the peer review.

## 5. Simulation Analysis

### 5.1. Transfer Function

Due to the barrel control system of water-cooled injection machines is really complex, it is difficult to model only by the mechanism. In this paper, several heating and cooling tests were carried out on the heating test-bed, and the heating and cooling curves of the cylinder under different heating power and cold circulating water conditions were obtained. Then, the transfer functions of heating and cooling devices in the process of cylinder temperature control are obtained by using the method of experimental modeling.

The transfer function of the heating device: the barrel is heated with the heating wire, and it gradually heats up. Using MATLAB software to fit the time data and temperature data collected at various moments, it is found that the curve is approximately S-shaped. The Ziegler–Nichols response curve method is used to prove that the transfer function of the heating device is approximately an order inertia lag link. Then, calculated by the Cohen–Kuhn formula, and the transfer function can be obtained as follows:

(2) $$\begin{array}{c} G_{1}\left(s\right)=\frac{16e^{-20s}}{26.3s+1}. \end{array}$$

The transfer function of the cooling device: first, the barrel is heated up to 180°C, and subsequently, it is cooled with the aid of cold circulating water. In this process, the time data and temperature data at different times are collected, and the collected data are fitted into curves using MATLAB software. After processing and analyzing the data, the transfer function of the cooling device is approximately an order inertia lag link. Then, calculated by the Cohen–Kuhn formula, the transfer function can be obtained as follows:

(3) $$\begin{array}{c} G_{2}\left(s\right)=\frac{20e^{-13s}}{105s+1}. \end{array}$$

### 5.2. Simulation Analysis

In order to verify the effectiveness and advancement of expert adjustable fuzzy control strategy in the temperature control system for injection machines, the simulation and comparison of PID control, fuzzy PID control, and expert adjustable fuzzy controller (EAFC) are carried out by using the software of Simulink. As the control object, the temperature of the barrel compression section is set 200°C, and the fixed parameters of PID controller is set as KP = 0.52, KI = 0.36, and KD = 1.4. The simulation result of the above three controllers is shown in Figure 6. It can be seen from the figure that the overshoot of PID controller, fuzzy PID controller, and EAFC is 11.3°C, 5.2°C, and 0.6°C, respectively, the time to reach the steady state is 185s, 175s, and 90s, respectively, and the response speed is 56s, 91s, and 90s, respectively. According to the analysis of the above data, EAFC has the advantages of small amount of overshoot and fast response speed.

In order to verify the robustness and anti-interference capability of EAFC, a negative interference signal of 20°C is added at 200s of simulation time, as shown in Figure 7. The maximum fluctuation amplitude of curves in PID controllers, fuzzy PID controllers, and EAFC are 29°C, 17.3°C, and 9.4°C, respectively, and the time required to reach the steady state is 110 s, 75s, and 53s, respectively. It shows that EAFC has great anti-interference ability and robustness.

Because of the great amount of complex interference factors in the control system of water-cooled injection machines, the control object model is easily mismatched. In order to verify EAFC has better robustness on the problems of model mismatching, on the basis of adding interference factors, the process gain and time constant of transfer function in the barrel temperature control system are, respectively, increased by 20% to be simulated and compared, which is shown in Figure 8. After model mismatch, the parameters of PID controllers, fuzzy PID controllers, and EAFC are shown in Table 4.

The article "Application of Expert Adjustable Fuzzy Control Algorithm in Temperature Control System of Injection Machines" was retracted in 2023. Reasons: unreliable results or conclusions; concerns about the data; concerns about the results or conclusions; concerns about the peer review.

As can be seen from Figure 8 and Table 4, when the process gain and time constant of transfer function in the barrel temperature control system are, respectively, increased by 20%, the overshoot, the time reach to steady state, and secondary steady state time have all increased. Obviously, EAFC is least affected by model mismatch and has the optimal robustness of model mismatch.

When the simulation time is 150 s, the input signal of the simulation control system is changed from 200°C to 100°C to verify the tracking performance of EAFC. As shown in Figure 9, when the simulation curve of the temperature control system deviates from the control target temperature under the influence of the interference input signal, the output curves of the three controllers appear in a transient unstable state. There is a large overshoot in the PID controller curve, and the response speed of the fuzzy PID controller is slower than that of EAFC. Generally speaking, EAFC play the best performance in tracking.

According to the simulation and comparison of Figures 6–9, EAFC is superior to PID controller and fuzzy PID controller in controller performance, anti-interference ability, the robustness of model mismatch, and tracking performance and has advantages and effectiveness in barrel temperature control of injection machines.

## 6. Conclusion

The temperature control system of water-cooled injection machines has the characteristics of complexity and nonlinearity, which is difficult to achieve good control effects using the traditional PID control. At the same time, by analyzing the limitations of fuzzy PID control due to the fixed fuzzy domain, the expert control rules are proposed to adjust the domain of fuzzy PID control. Then, EAFCA is designed to improve the stability and accuracy of the barrel temperature control system of injection machines. The simulation results show that EAFCA has the advantages of small overshoot, fast adjusting speed, strong anti-interference ability, good robustness of model mismatch, and good tracking ability, which can meet the requirements of the barrel temperature control. By taking CPU315–2PN/DP PLC and industrial PC as the core of hardware, the control system of DCS for injection machines is established. Based on the platform of Step7 and WinCC software, the human-machines reaction interface is developed. Finally, the barrel temperature control system of injection machines has been upgraded well.

The article "Application of Expert Adjustable Fuzzy Control Algorithm in Temperature Control System of Injection Machines" was retracted in 2023. Reasons: unreliable results or conclusions; concerns about the data; concerns about the results or conclusions; concerns about the peer review.

## Figures and Tables

**Figure 1:** Schematic diagram of temperature control of the injection molding machine.

**Figure 2:** The barrel temperature control system adopting expert-adjustable fuzzy-domain PID controller for injection machines.

**Figure 3:** The hardware configuration diagram of DCS.

**Figure 4:** Temperature control flow chart of injection machines.

**Figure 5:** Temperature control flow chart of injection machines.

**Figure 6:** Performance simulation comparison of the three controllers.

**Figure 7:** Simulation diagram of anti-interference ability comparison of three controllers.

**Figure 8:** Simulation and comparison of process gain and time constant increased by 20%.

**Figure 9:** Simulation and comparison of tracking performance of three controllers.

**Table 1:** Parameters of the fuzzy PID controller.

Variables	e	ec	Δ*K*_*P*_	Δ*K*_*I*_	Δ*K*_*D*_
Linguistic variable	e	ec	Δ*K*_*P*_	Δ*K*_*I*_	Δ*K*_*D*_
Basic domain	[−5,5]	[−3,3]	[−0.8,0.8]	[−0.5,0.5]	[−10,10]
Fuzzy subsets	{NB, NM, NS, *Z*, PS, PM, PB}				
Fuzzy domain	[−6,6]	[−6,6]	[−0.8,0.8]	[−0.05,0.05]	[−6,6]
Quantization factor	4.2	2	1	1	0.6
Membership function	Triangle				

**Table 2:** The rules table of fuzzy PID correction parameters Δ*K*_*P*_, Δ*K*_*I*_, and Δ*K*_*D*_.

e	ec						
	NB	NM	NS	Z	PS	PM	PB
NB	PB/Z/PS	PB/Z/PS	PM/PM/Z	PM/Z/NS	PS/Z/NS	PS/NS/NM	PS/NS/PM
NM	PM/Z/NS	PM/Z/NS	PS/NM/NS	PS/NM/NS	Z/NS/NS	Z/Z/PS	NS/Z/PS
NS	PM/Z/NB	PS/Z/NB	PS/NS/NS	Z/NS/NS	Z/Z/Z	NS/Z/PS	NM/PS/Z
Z	PS/Z/NS	PS/Z/NS	Z/NS/NS	Z/Z/Z	NS/PS/Z	NS/Z/Z	NM/Z/PS
PS	Z/Z/NM	Z/Z/NM	Z/Z/NS	NS/PS/NS	NS/PS/Z	NM/Z/PS	NM/PM/Z
PM	PM/Z/NS	PS/Z/NS	PS/PS/NS	PM/PM/PS	PS/PM/PS	PM/Z/PS	PB/Z/PS
PB	PB/Z/PS	PS/Z/Z	NS/PM/PS	PS/PM/PS	PM/PM/PM	PM/PS/PM	PB/Z/PS

**Table 3:** Hardware selection list of the DCS.

Number	Name of the hardware	Hardware parameters	Hardware model	Quantity
1	CPU315-2PN/DP	2PN, 1DP, 8M micro-memory card	6ES7315-2EH14-0AB0	1
2	160 guide	Module installation	6ES7390-1AB60-0AA0	1
3	PS307	AC120/230V, 5 A	6ES7307-1BA01-0AA0	1
4	HMI	KTP1000 basic color PN	6AV6447-0AF11-3AX0	1
5	SM321	16DI, 24VDC, potential isolation, front connector	6ES7321-1BH02-0AA0	2
6	SM322	16DO, 0.5 A, potential isolation, front connector	6ES7322-1BH01-0AA0	2
7	SM331	8AI, 13 bit, 66 ms, potential isolation, front connector	6ES7331-1KF02-0AB0	1
8	SM332	8AO, 11/12 bit, potential isolated, front connector	6ES7332-4JB51-0AB0	1
9	SM331	8AI, PT100/200/300, front connector	6ES7331-7PF02-0AB0	1
10	Temperature sensor	-200-250°C, 3.2 mm, ±0.05°C	PT100	4
11	Solenoid valve	0.5–50 bar, normally closed, 4-20 mA	JGZBM	3
12	Industrial PC	16G, 1T, 2G dependent display, i7	DELL	1
13	SSR	220VAC, 50A	ZHIHE	6

The article "Application of Expert Adjustable Fuzzy Control Algorithm in Temperature Control System of Injection Machines" was retracted in 2023. Reasons: unreliable results or conclusions; concerns about the data; concerns about the results or conclusions; concerns about the peer review.

**Table 4:** The parameters in three controllers with process gain and time constant increased by 20%.

The controller	Overshoot/°C	Rise time/s	Steady state time/s	Interference amplitude/°C	Secondary steady state time/s
PID	34.5	43	180	35.5	140
The fuzzy PID	7.5	82	165	20	110
EAFCA	1.3	81	125	9.2	60

## Data Availability

The data used to support the findings of this study are available from the corresponding author upon request.
